The article "Diagnostic Markers and Molecular Dysregulation Mechanisms in the Retinal Pigmented Epithelium and Retina of Age-Related Macular Degeneration" was published in 2022. Journal: J Healthc Eng.

# Diagnostic Markers and Molecular Dysregulation Mechanisms in the Retinal Pigmented Epithelium and Retina of Age-Related Macular Degeneration

**DOI:** 10.1155/2022/3787567

**Published:** 2022-02-10

**Authors:** Yao Li, Jing Fu, Jiawen Liu, Huayin Feng, Xueyi Chen

**Affiliations:** ^1^Department of Ophthalmology, The First Affiliated Hospital of Xinjiang Medical University, Urumqi 830054, Xinjiang, China; ^2^Jiangmen Central Hospital, Jiangmen 529000, Guangdong, China

## Abstract

Age-related macular degeneration (AMD) is a chronic and progressive macular degeneration disease, which can also lead to serious visual loss. In our research, we aim to efficiently identify biomarkers relevant for AMD diagnosis. We collected the gene expression data of retinal segmented epithelium (RPE) and retina tissues of GSE29801 and GSE135092 and performed differential expression analysis. The differentially expressed genes (DEGs) related to the RPE and retina in the two sets of data were identified and enriched by intersection analysis. A PPI network was constructed for intersection genes, and the top 20 genes with the largest connectivity in the network were selected as candidate genes. The LASSO model was used to identify key genes from candidate genes, and the nomogram and ROC curve were used to evaluate the diagnostic ability of key genes. We identified 464 intersection genes associated with RPE and 509 intersection genes associated with retina. The TGF-beta signaling pathway was enriched by RPE-related DEGs, while oxidative phosphorylation was enriched by retina-related DEGs. Among the candidate genes of RPE, the LASSO model identified 7 key genes. MAPK1 and LUM can predict the clinical diagnosis of AMD. Among the candidate genes of retina, the LASSO model identified four key genes. PTPN11 has the highest predictive diagnostic value. The results suggest that the imbalance mechanism of RPE in AMD may be related to the TGF-beta signaling pathway, and the imbalance mechanism of the retina may be related to oxidative phosphorylation. MAPK1 and LUM are potential diagnostic markers of RPE, and PTPN11 is a potential diagnostic marker of the retina. Also, our results provide a theoretical basis for better understanding the molecular mechanisms of AMD onset and treatment in the future.

## 1. Introduction

Age-related macular degeneration (AMD) is a chronic and progressive macular degenerative disease. Its pathogenesis is mainly caused by the retention of disk membranes due to the reduced phagocytic ability of the retinal pigment epithelium [1]. It has been reported that AMD is the third most blinding eye disease worldwide, and its incidence is second only to cataract and refractive error [2–4]. According to the global burden of disease study, the number of people with AMD will increase substantially in the next decades as the global population ages [5]. Experts have predicted that there will be approximately 196 million patients with AMD worldwide in 2020, and by the end of 2040, the number of global patients with ADM will increase to 288 million [6, 7]. Therefore, there is an urgent need for relevant clinical markers to assist clinicians to make an accurate early diagnosis of AMD and predict clinical outcomes without individualized medical treatment provision.

Fundus color illumination, optical coherence tomography, vascular imaging with optical coherence tomography, and fundus angiography are commonly used in the clinic to identify and predict early, intermediate, and late AMD progression, as well as to predict AMD recurrence and prognosis. But, until now, there is still no consensus to systematically identify and predict AMD biomarkers, so for the research of AMD, further exploration is needed. The onset of AMD has a certain complexity and is triggered by a combination of genetic and environmental factors [8, 9]. The study of AMD prediction from the genetic level may become one of the important methods for AMD diagnosis and treatment in the future.

There are currently many studies on the search for biomarkers to assist in the early diagnosis of AMD patients. Some studies propose that earlier relevant genetic testing of populations is able to play an important role in AMD prediction [10–13]. However, even though an increasing number of AMD-related genes are currently being discovered, the mechanism of their occurrence has failed to get a clear explanation. Previous studies have also estimated risk scores for AMD by building models based on different factors [14, 15]. But, since the occurrence of AMD is a complex process, many pathways including the complement pathway, lipid metabolism, angiogenesis, and many related genes may be involved [16–22]. Therefore, it is difficult to establish a prediction model for AMD, and it still needs deep research.

To efficiently identify biomarkers relevant for AMD diagnosis, we proposed a systematic pipeline for identifying relevant genes for AMD by collecting gene expression data of the retinal pigment epithelium (RPE) and retina in gse29801 and gse135092 and performing bioinformatics analysis. This method has high predictive value for early clinical diagnosis of AMD and provides a theoretical basis for better understanding the molecular mechanisms of AMD onset and treatment in the future.

## 2. Materials and Methods

### 2.1. Methods

The lesions of AMD show long-term progressive dynamic development, and according to the 2019 American Academy of ophthalmology clinical guidelines, AMD is divided into no AMD, early AMD, intermediate AMD, and advanced AMD [23]. Usually, early AMD patients are asymptomatic [24] and, thus, easily ignored, while after that, AMD macular lesions can skip to progress into map like atrophy or wet AMD, which leads to macular atrophy and scarring and, finally, blindness. Although, in recent years, the advent of antivascular endothelial growth factor drugs, which have contributed to a delay in the development of AMD, has not been able to solve the problem fundamentally [25]. Therefore, the early screening of indicators with predictive value using various methods and their application in the initial screening, disease warning, and clinical treatment guidance of AMD is beneficial for the early diagnosis and precision treatment of AMD, which is of great significance to prevent the occurrence of AMD and the vision loss of patients.

Studies have shown that TGF-*β* mediated signaling pathways play an important role in ocular diseases [26]. Radeke et al. [27] also found that targeted inhibition of TGF-*β* signaling may be an effective way to delay the progression and the production of large numbers of RPE cells. In addition, we also found that oxidative phosphorylation (OXPHOS) was enriched by retina-associated DEGs. The retinal pigment epithelium is very active in metabolism and consists of a large number of mitochondria [28]. In the process of OXPHOS, the form of ATP and reactive oxygen species was produced from these organelles and considered cellular energy [29].

### 2.2. Data Processing

The data used in this study were downloaded from the Gene Expression Omnibus (GEO) database. GSE29801 included gene expression profiles of RPE and retina tissue samples from 31 controls and 26 AMD patients. GSE135092 included gene expression profiles of RPE and retina tissue samples from 99 controls and 23 AMD patients. The differential expression analysis between AMD and controls for the RPE or retina in GSE29801 was performed using limma package [30]. For GSE135092, the differential expression analysis was performed using DESeq2 package [31]. Significantly differentially expressed genes (DEGs) were screened with *P* < 0.05.

### 2.3. Enrichment Analysis

Gene Ontology (GO) and Kyoto Encyclopedia of Genes and Genomes (KEGG) pathway enrichment analysis of DEGs were carried out by the clusterProfiler package [32]. Significantly enriched terms in GO and KEGG pathways were screened by setting the criterion of *P* < 0.05.

### 2.4. Protein-Protein Interaction (PPI) Network

The PPI network of DEGs was constructed based on the Search Tool for the Retrieval of Interacting Genes (STRING) (http://string-db.org/) database. The top 20 genes with the most connectivity were filtered out as candidate genes for subsequent analysis. The PPI network was visualized by Cytoscape software.

### 2.5. Logistic Regression Analysis

The logistic regression analysis was used to construct a forest plot for candidate genes. Then, a binomial least absolute shrinkage and selection operator regression (LASSO) model was built based on candidate genes using the glmnet R package [33]. The key genes were identified according to the optimal lambda. A nomogram was used to display the results of the logistic analysis including all key genes. The R packages' rms was used to construct the nomogram. The receiver operating characteristic (ROC) curve was plotted, and the area under the ROC curve (AUC) was calculated with “pROC” package [34].

## 3. Results

### 3.1. Differentially Expressed Genes in AMD

To identify aberrantly expressed genes in AMD patients, we performed differential analysis between RPE, retina, and controls separately. In GSE29801, we identified 2675 DEGs for the RPE (Figure 1(a)) and 2415 DEGs for the retina (Figure 1(b)). In GSE135092, we identified 4426 DEGs for the RPE (Figure 1(c)) and 6900 DEGs for the retina (Figure 1(d)). Through intersection analysis, we identified 464 intersection genes and considered RPE-associated DEGs (Figures 2(a) and 2(b)) and 509 intersection genes and considered retina-associated DEGs (Figures 2(c) and 2(d)).

### 3.2. Biological Function Enrichment Analysis

To identify the molecular dysregulation mechanism of the RPE and retina in AMD patients, we performed enrichment analysis of intersection genes. For the biological processes (BPs) in RPE, intersection genes were enriched in negative regulation of cell differentiation, negative regulation of cell population proliferation, and regulation of epithelial to mesenchymal transition (Figure 3(a)). The TGF-beta signaling pathway, Hippo signaling pathway, and Wnt signaling pathway were found in KEGG pathways of RPE (Figure 3(b)). On the other hand, positive regulation of the G protein-coupled receptor signaling pathway, aerobic electron transport chain, and mitochondrial ATP synthesis coupled electron transport in BPs were significantly enriched by intersection genes of the retina (Figure 3(c)). KEGG signaling pathways in the retina were mainly included oxidative phosphorylation, pathways of neurodegeneration, and phagosome (Figure 3(d)).

### 3.3. PPI Network Construction for the RPE and Retina

To identify genes with significant influence in the RPE and retina, we constructed a PPI network for the intersection genes separately. By identifying the degree of connectivity among the genes in the network, we obtained the top 20 genes with the largest degree of connectivity as candidate genes. Finally, we identified PPARG, MAPK1, WNT2, THBS2, LUM, BMP7, DKK1, FMOD, CHEK2, NCAN, SREBF1, SCD, SFRP1, GATA2, CEBPA, PTPRZ1, ADAMTS4, COL5A2, TGFB2, and SNAI1 in RPE (Figure 4(a)). HSP90AA1, RPL4, MRPS7, HSPE1, CCT7, RPL23A, CCT4, NDUFAB1, MRPL4, MRPS15, RPL15, PA2G4, SOD1, TLR4, RPL29, CYC1, MRPL2, CARS, PTPN11, and MRPS12 were identified in the retina (Figure 4(b)). The results of logistic regression analysis showed that candidate genes may serve as protective or risk factors contributing to AMD in the RPE (Figure 4(c)) and retina (Figure 4(d)).

### 3.4. Identification of Key Genes for the RPE and Retina

Furthermore, we performed LASSO regression analysis for candidate genes in RPE and retina, respectively. The number of independent coefficients gradually decreases with increasing lambda (Figure 5(a)). Therefore, we selected the model with the best lambda of 0.01933388 as the final model, containing a total of 7 signatures (SREBF1, MAPK1, SFRP1, WNT2, PTPRZ1, LUM, and THBS2) in the RPE (Figure 5(b)). For the retina, we selected the model with the best lambda of 0.02094517 as the final model, which contained a total of 4 signatures (HSP90AA1, HSPE1, SOD1, and PTPN11) in the retina (Figures 5(c) and 5(d)). These signatures were then considered as key genes of the RPE or retina.

To further evaluate the diagnostic role of the key genes, a nomogram was constructed using logistic repression analysis. Of which, RPE, MAPK1, and LUM contributed the most to the risk of AMD (Figure 6(a)). PTPN11 contributed the most to the risk of the retina in AMD (Figure 6(b)). The AUC values of MAPK1 and LUM were 0.675 and 0.787 (Figure 6(c)), and the AUC value of PTPN11 was 0.684 (Figure 6(d)). These data suggested that key genes may predict AMD diagnosis, especially MAPK1 and LUM for RPE and PTPN11 for the retina.

## 4. Discussion

We collected and analyzed gene expression data from RPE and retina tissues, leading to the identification of aberrantly expressed genes in AMD patients. The analysis results suggested that the TGF-*β* signaling pathway was enriched by RPE-associated DEGs. TGF-*β* is synthesized and secreted in various tissues of the posterior segment of the eye, such as the cornea, iris, lens epithelial cells, trabecular meshwork cells, ciliary body epithelial cells, and retinal pigment epithelial cells, and it plays important roles in cell growth and differentiation [35]. Reactive oxygen species may damage mitochondrial DNA, and then, damaged mitochondrial DNA leads to mitochondrial dysfunction and increased ROS production, which initiates a vicious cycle [36]. The retinal pigment epithelium is particularly vulnerable to mitochondrial dysfunction and ROS damage and does not regenerate [37, 38]. The high prevalence of AMD in the elderly may be related to this.

Among the candidate genes of RPE, MAPK1 and LUM were predictive for the clinical diagnosis of AMD, and their AUC values reached 0.675 and 0.787. Mitogen-activated protein kinase 1 (MAPK1) is an important protein in MAPK signaling, which acts as a negative regulator of MAPK signaling and regulates cell proliferation and growth [39]. Kyosseva [40], through investigation studies, considered an association between MAPK signal transduction and AMD in humans and animals and suggested that the use of specific MAPK inhibitors may be a potential treatment for AMD. In contrast, the lumican (LUM) gene has been studied by Chinese scholars in the field of high myopia or pathological myopia [41–43] and is an important factor in maintaining the biomechanical properties of the sclera [44]. Among the retina's candidate genes, protein tyrosine phosphatase non-receptor type 11 (PTPN11) had the highest diagnostic predictive value, reaching an AUC value of 0.684. The PTPN11 gene is a mutation-prone gene with a large number of mutations and genetic variations associated with human diseases. Reports on PTPN11 have focused on the development and prognosis of diseases such as promyelocytic leukemia [45, 46], myelodysplastic syndrome in children [46], ulcerative colitis [47], and gastric cancer [48]. At present, we have not retrieved any conclusion from the study that PTPN11 and LUM have a significant association with AMD, so they may be new markers for AMD. Although investigation studies investigating the association between AMD are currently missing for the abovementioned genes, MAPK1 and LUM, in addition to PTPN11, all play a role in different ocular diseases.

## 5. Conclusions

In conclusion, our study efficiently identified biomarkers relevant for AMD diagnosis. Furthermore, we proposed a systematic pipeline for identifying relevant genes for AMD and performed bioinformatics analysis. Our finding has high predictive value for early clinical diagnosis of AMD in the future. However, there are still some shortcomings in our research. This study did not carry out specific investigation for the population and did not consider the influence of environmental factors in the occurrence and development of AMD, and the expression of key genes in AMD was not experimentally verified, but the findings also provide a new idea for future clinical AMD early diagnosis and prevention research. To clarify the association between the abovementioned genes and AMD, follow-up can be clarified through population-based epidemiological and gene level investigations.

## Figures and Tables

**Figure 1:** Identification of DEGs in AMD. (a) Volcano plot of DEGs between AMD and controls in RPE of GSE29801. (b) Volcano plot of DEGs between AMD and controls in the retina of GSE29801. (c) Volcano plot of DEGs between AMD and controls in the RPE of GSE135092. (d) Volcano plot of DEGs between AMD and controls in retina of GSE135092. Red represents upregulation, and blue represents downregulation.

**Figure 2:** Intersection analysis of DEGs. (a) Intersection of DEGs in RPE of GSE29801 and GSE135092. (b) Expression heatmap of intersection genes in RPE. Red represents upregulation, and blue represents downregulation in AMD. (c) Intersection of DEGs in the retina of GSE29801 and GSE135092. (d) Expression heatmap of intersection genes in the retina. Red is upregulated, and blue is downregulated in AMD. AMD, age-related macular degeneration.

**Figure 3:** Enrichment analysis of intersection genes in the RPE and retina. (a) The main GO terms enriched by intersection genes of RPE. (b) The main KEGG pathways enriched by intersection genes of RPE. (c) The main GO terms enriched by intersection genes of the retina. (d) The main KEGG pathways enriched by intersection genes of the retina.

**Figure 4:** Identification and evaluation of candidate genes in the RPE and retina. (a) The top 20 genes with most connectivity in the PPI network of the RPE. (b) The top 20 genes with most connectivity in the PPI network of the retina. (c) The forest plot of candidate genes of the RPE. (d) The forest plot of candidate genes of the retina.

**Figure 5:** Identification of key diagnostic genes for AMD. (a) LASSO coefficient profiles of candidate genes in the RPE. (b) Selection of optimal parameter (*λ*) in the LASSO model of the RPE. (c) LASSO coefficient profiles of candidate genes in the retina. (d) Selection of optimal parameter (*λ*) in the LASSO model of the retina.

**Figure 6:** Diagnostic predictive power of key genes. (a) Nomogram of key genes of the RPE to predict the risk for AMD. (b) Nomogram of key genes of the retina to predict the risk for AMD. (c) ROC curve analyses based on the key genes of the RPE. (d) ROC curve analyses based on the key genes of the retina.

## Data Availability

The datasets used and/or analyzed during the current study are available from the corresponding author on reasonable request.
